# 5-Year Survivorship and Outcomes of Robotic-Arm-Assisted Medial Unicompartmental Knee Arthroplasty

**DOI:** 10.1155/2022/8995358

**Published:** 2022-05-06

**Authors:** Michael A. Gaudiani, Linsen T. Samuel, John N. Diana, Jennifer L. DeBattista, Thomas M. Coon, Ryan E. Moore, Atul F. Kamath

**Affiliations:** ^1^Department of Orthopaedic Surgery, Henry Ford Hospital, 2799 W Grand Blvd. K12 Detroit MI 48202, USA; ^2^Department of Orthopaedic Surgery, Cleveland Clinic Foundation, 9500 Euclid Avenue, Mail Code A40, Cleveland, Ohio 44195, USA; ^3^Coon Joint Replacement Institute, 6 Woodland Road Suite 202, St. Helena, California 94574, USA

## Abstract

**Purpose:**

While unicompartmental knee arthroplasty (UKA) has demonstrated benefits over total knee arthroplasty (TKA) in selected populations, component placement continues to be challenging with conventional surgical instruments, resulting in higher early failure rates. Robotic-arm-assisted UKA (RA-UKA) has shown to be successful in component positioning through preop planning and intraop adjustability. The purpose of this study is to assess the 5-year clinical outcomes of medial RA-UKA.

**Methods:**

This study was a retrospective review of a single-center prospectively maintained cohort of 133 patients (146 knees) indicated for medial UKA from 2009 to 2013. Perioperative data and 2- and 5-year Knee injury Osteoarthritis Outcome Score (KOOS), Western Ontario and McMaster Universities Osteoarthritis Score (WOMAC), and Forgotten Joint Score (FJS) outcome measures were collected. Five-year follow-up was recorded in 119 patients (131 knees).

**Results:**

Mean follow-up was 5.1 ± 0.2 years. Mean age and BMI were 68.0 ± 8.1 years and 29.3 ± 4.7 kg/m^2^, respectively. At 2-year follow-up, mean KOOS, WOMAC, and FJS were 71.5 ± 15.3, 14.3 ± 7.9, and 79.1 ± 25.8, respectively. At 5-year follow-up, mean KOOS, WOMAC, and FJS were 71.6 ± 15.2, 14.2 ± 7.9, and 80.9 ± 25.1, respectively. Mean change in KOOS and WOMAC was 34.6 ± 21.4 and 11.0 ± 13.6, respectively (*p* < 0.001 and *p* < 0.001). For patient satisfaction at last follow-up, 89% of patients were very satisfied/satisfied and 5% were dissatisfied. For patient activity expectations at last follow-up, 85% met activity expectations, 52% were more active than before, 25% have the same level of activity, 23% were less active than before, and 89% were walking without support. All patients returned to driving after surgery at a mean 15.2 ± 9.4 days. Survivorship was 95% (95% CI 0.91-0.98) at 5 years. One knee (1%) had a patellofemoral revision, two knees (1.3%) were revised to different partial knee replacements, and five knees (3.4%) were converted to TKA.

**Conclusion:**

Overall, medial RA-UKA demonstrated improved patient-recorded outcomes, high patient satisfaction, met expectations, and excellent functional recovery. Midterm survivorship was excellent. Longitudinal follow-up is needed to evaluate long-term outcomes of robotic-arm-assisted UKA procedures.

## 1. Introduction

Unicompartmental knee arthroplasty (UKA) is an increasingly popular and reliable surgical solution for isolated medial knee osteoarthritis with positive clinical outcomes and excellent survivorship [1–3]. Many consider UKA a superior option to total knee arthroplasty (TKA) as UKA has multiple advantages including faster recovery [4], better range of motion [5], fewer complications [6], and easier revisions [7]. Despite these advantages, UKA is a technically demanding procedure with reported failures due to iatrogenic surgical factors including lower limb postoperative malalignment and component malpositioning [8]. Additionally, recent registry data reports UKA has a higher revision rate and lower annual survivorship when compared to TKA [3, 9].

To better optimize UKA survivorship, robotic-arm-assisted UKA (RA-UKA) was developed to improve surgeon reliability and reproducibility of the procedure. RA-UKA allows for improved soft-tissue balancing, reproducible leg alignment, and accurate implant position [10–14]. In comparison to conventional manual UKA, RA-UKA has been shown to have comparable functional outcomes [15] and improved component positioning and reliability [16, 17]. As recently reported in the literature, RA-UKA has fewer revisions and higher patient satisfaction compared to conventional UKA [18] as well as excellent short-term survivorship [19]. While short-term and midterm survivorship and satisfaction have been positive for RA-UKA [19–21], there is still a need for midterm follow-up data regarding patient-recorded outcomes (PROMs), satisfaction, and survivorship following RA-UKA to better assess the clinical outcomes using a modern robotic arthroplasty system.

Therefore, the purpose of our study was to review the PROMs, survivorship, and satisfaction following RA-UKA at a single center at 5-year follow-up. Our hypothesis is that RA-UKA at 5-year follow-up will have positive PROMs, excellent survivorship, and high satisfaction.

## 2. Methods

This study was a retrospective review of a single-center prospectively maintained cohort of 133 consecutive patients (146 knees) indicated for medial UKA from 2009 to 2013. Institutional review board approval was obtained at the institution in order to collect and analyze this data. Inclusion criteria included all patients over 21 years of age who required primary medial UKA. These patients failed nonoperative management of their joint disease and were candidates for partial joint replacement because of pain and joint stiffness that interfered with their performance of normal daily activities. Exclusion criteria included patients needing lateral RA-UKA, patients with active infection, patients with not enough bone stock to allow for insertion and fixation of the components, patients with insufficient soft tissue integrity to allow for stability, patients with neurological or muscular deformity that did not allow for control of the knee, patients unable cognitively to complete health-related quality of life forms, and pregnant women. Lateral compartment RA-UKA was excluded due to the different osteoarthritis etiologies, surgical indications, and intraoperative component positioning. All patients enrolled had radiographic evidence of osteoarthritis in the medial compartment and received the Restoris MCK (Mako Surgical Corp. (Stryker), Fort Lauderdale, FL) UKA implant. All surgeries were performed with robotic assistance Mako System (Mako Surgical Corp. (Stryker), Fort Lauderdale, FL).

Data was collected by a research coordinator. Patient questionnaires were given to patients at their office visit. For patients that did not come in for visits, they were sent via regular mail or email by the research coordinator. Patients were asked if revision surgery took place. If the patients answered no, the patient was asked to rate their overall satisfaction with their operated knee on a 5-item Likert scale: “very satisfied,” “satisfied,” “neutral,” “dissatisfied,” or “very dissatisfied.” Before they were considered lost to follow-up, phone contact for each patient was attempted three times. Intraoperative data collected included tourniquet time, total operating room time, and estimated blood loss. At discharge, patient distance walked and pain score were collected.

Five-year and two-year postoperative follow-up was recorded in 119 patients (131 knees), 71 left knees and 60 right knees. Data collected at all follow-up timepoints included demographic information (date of birth, date of surgery, body mass index (BMI), and laterality), patient satisfaction with Mako operative knee, patient activity expectation, support with walking, and patient-recorded outcome measures (PROMs). PROMs collected were the reduced Knee injury Osteoarthritis Outcome Score (KOOS), reduced Western Ontario and McMaster Universities Osteoarthritis Score (WOMAC), and Forgotten Joint Score (FJS). The reduced WOMAC is a truncated version of the WOMAC which is designed to assess pain, disability, and joint stiffness in the OA patient. The reduced KOOS assesses the patient's opinion regarding their knee and its associated OA. Poor outcomes are reported with a lower score and good outcomes with a higher score. The FJS determines how aware the patient is of their joint in their everyday life. Substantial clinical benefit (SCB) and minimal clinically improvement difference (MCID) threshold used for KOOS scoring was 20 and 14, respectively [22]. WOMAC MCID threshold used was 10 [23]. Patient acceptable symptom state (PASS) threshold used for the FJS score was 40.63 [24].

Descriptive statistical analysis and Student *t*-tests of demographics and patient-recorded outcome scores were performed on Microsoft Excel Version 16.16 (Microsoft Inc., Redmond, WA). Kaplan-Meier survivorship was calculated using GraphPad Prism 8.0.0 (GraphPad Software Inc., San Diego, CA).

## 3. Results

Mean follow up was 5.1 ± 0.2 years (range, 4.96 to 6.00). Mean age and BMI were 68.0 ± 8.1 years (range, 46.9 to 88.2) and 29.3 ± 4.7 kg/m^2-^ (range, 18.5 to 46.7), respectively. Intraoperatively, mean estimated blood loss was 12.0 ± 8.5 ml (range, 0 to 30); mean tourniquet time was 31.4 ± 9.7 minutes (range, 3 to 61), and mean total operative time was 104.3 ± 67.4 minutes (range, 10 to 847). At time of discharge, mean distance walked was 266 ± 58.3 feet (range, 100 to 450), mean pain score was 2.3 ± 2.3 (range, 0 to 8), and mean hemoglobin was 11.8 ± 1.1 mg/dl (range 9.1 to 14.4).

Preoperative mean KOOS and WOMAC were 43.1 ± 11.2 (range, 20 to 74.4) and 72.8 ± 12.8 (range, 53 to 100). At 2-year follow-up, mean KOOS, WOMAC, and FJS were 71.5 ± 15.3 (range, 33.1 to 90.0), 85.7 ± 7.9 (range, 50 to 100), and 79.1 ± 25.8 (range, 0 to 100), respectively. At 5-year follow-up, mean KOOS, WOMAC, and FJS were 71.6 ± 15.2 (range, 32.5 to 90), 85.8 ± 7.9 (range, 59 to 100), and 80.9 ± 25.1 (range 2 to 100), respectively (Table 1). WOMAC MCID was met in 64% of patients, and KOOS MCID and SCD was met in 86% and 78%, respectively. Mean change in KOOS and WOMAC was 34.6 ± 21.4 and 11.0 ± 13.6, respectively (*p* < 0.001 and *p* < 0.001). For patient satisfaction at last follow-up, 89% of patients were very satisfied/satisfied and 5% were dissatisfied. For patient activity expectations at last follow-up, 85% met activity expectations; 52% were more active than before; 25% have the same level of activity; 23% were less active than before; and 89% were walking without support. All patients returned to driving after surgery at a mean of 15.2 ± 9.4 days (range, 1 to 41). Survivorship was 95% (95% CI 0.91-0.98) at 5 years. One knee (1%) had a patellofemoral revision, two knees (1.3%) were revised to different partial knee replacements, and five knees (3.4%) were converted to TKA.

## 4. Discussion

The purpose of this study was to assess the PROMs, patient satisfaction, and survivorship at 5-year follow-up of a single center's experience with RA-UKA for medial osteoarthritis. We found positive and significant improvement in PROMs, excellent survivorship, and high patient satisfaction with medial RA-UKA. This confirmed out hypothesis that medial RA-UKA would be successful at 5-year follow-up.

In our study, we found predominantly good to excellent PROM results with significant improvement from preoperative values at 5-year follow-up. Burger et al. performed a similar analysis of 713 medial RA-UKA at 4.9-year follow-up and reported a mean KOOS of 84.3 [25]. While our KOOS scores were lower, both studies reported similar good to excellent KOOS results. Our cohort was on average older (68.0 years vs. 63.5 years) which could explain our lower results as older age has been associated with lower KOOS scores postoperatively in subgroup analysis [19]. At short-term follow-up, Zambianchi et al. also reported good to excellent KOOS scores (mean 85.5) following medial RA-UKA in a slightly younger cohort (mean 65.4 years) than the present study [19]. Additionally, both our KOOS and WOMAC results are above the MCID and SCB thresholds indicating that our significant improvement in KOOS and WOMAC is associated with clinical benefit. Overall, the positive results of our PROMS indicate that at 5-year follow-up RA-UKA is on average restoring knee function and improving quality of life.

Our FJS scores (mean 80.9) indicate that at 5-year follow-up on average patients undergoing medial RA-UKA are less aware of their artificial knee in comparison to normative values of the United States population (median 75.0) [26]. The FJS score has a benefit compared to the other PROMs used in that it does not have a ceiling effect and can better differentiate between good and excellent results. Our mean FJS was higher than values seen in conventional UKA (mean 68.9) [27] and in TKA at 2-year follow-up (mean 59.8) as well as above the PASS threshold [28]. Zuiderbaan et al. directly compared a cohort of RA-UKA and TKA and similarly found that RA-UKA was more likely forgotten compared to TKA [28]. The difference is likely due to more bone and soft tissue conservation seen with RA-UKA versus TKA.

Our study reported an excellent survivorship at 5-year follow-up of 95% which is similar to the reported values seen in the literature. Burger et al. recently reported the five-year survivorship of medial RA-UKA to be 97.8%, and Kleeblad et al. reported 97.5% survivorship at midterm follow-up [21, 25]. As expected, improved survivorship is also seen in shorter follow-up studies with Zambianchi et al. reporting 99% [19], Dretakis and Igoumenou reporting 100% [29], and Pearle et al. reporting 98.8% [20] for medial RA-UKA. Conventional UKA has also been recently found to have similar high survivorship of 97.2% and 97.7% at 5-year follow-up [30, 31]. While these results are comparable to RA-UKA, both studies are from experienced surgeons and high volume centers. Their excellent survivorship is likely not reproducible at low volume centers as they have been shown to have higher revision rates [32, 33]. This is reflected in recent registry data where conventional UKA has a higher revision rate compared to RA-UKA at three-year follow-up [3]. Overall, our study reports excellent survivorship of RA-UKA which is at least comparable to conventional UKA. More research is needed directly to compare the long-term outcomes of these surgeries.

The vast majority of our patients had high satisfaction with their RA-UKA at 5-year follow-up. Our results are similar to what is reported in the literature. Kleeblad et al. reported on 432 knees at 5.7-year follow-up and found that 91% of patients were very satisfied or satisfied with their medial RA-UKA. Another study at average 4.25-year follow-up found that 96% of patients were very satisfied or satisfied with their medial RA-UKA [29]. In our study, RA-UKA had a higher patient satisfaction percentage compared to satisfaction seen historically in TKA patients (82% to 89%) [34]. The high patient satisfaction and overall positive outcomes of RA-UKA are likely due to the increased accuracy of component placement and optimal lower limb alignment.

Our study also reported lower estimated blood loss compared to TKA and longer operative time compared to conventional UKA and TKA. We found our blood loss to be minimal and much less in comparison to commonly accepted numbers for perioperative blood loss in TKA of 0.5 L to 1.5 L [35, 36]. This is concurrent with other studies and is due to the less invasive nature of the surgery [37]. The mean overall operative time was slightly longer than times reported for TKA and conventional manual UKA [38, 39]. Significantly longer operative times for RA-UKA have also been seen in other reports comparing RA-UKA and manual UKA with no difference in component placement accuracy, estimated blood loss, and intraoperative complications [40]. More research is necessary to determine the clinical significance of the longer operative time, and this must be weighed against the potential benefits of robotic assistance.

The present study has several limitations. First, we lack comparison cohorts of manual UKA and/or TKA; therefore, conclusions regarding the use of RA-UKA versus manual UKA and RA-UKA versus TKA are outside the scope of this study. Second, the senior authors are also very experienced with RA-UKA; therefore, patient selection and surgical technique are most likely optimized and it is unclear whether these results are reproducible for a less experience surgeon. Third, we do not report knee alignment parameters; therefore, we cannot make conclusions regarding the alignment of our patients; however, previous studies have demonstrated the accuracy of RA-UKA. Lastly, we also do not report in-depth analysis regarding the revisions in our cohort; therefore, we are not able to discern patient characteristics or traits that impact the likelihood of revision. This is an area for future research and would likely require more patients given our small number of revisions.

## 5. Conclusion

Overall, medial RA-UKA demonstrated improved patient-recorded outcomes, high patient satisfaction, and excellent survivorship at 5-year follow-up. Longitudinal follow-up is needed to evaluate long-term outcomes of robotic-arm-assisted UKA procedures.

## Figures and Tables

**Table 1:** Patient-recorded outcome measures of medial robotic-assisted UKA.

	Preop	2 year	5 years	Change	*p* value^a^
KOOS	43.1 ± 11.2	71.5 ± 15.3	71.6 ± 15.2	34.6 ± 21.4	<0.001
WOMAC	72.8 ± 12.8	85.7 ± 7.9	85.8 ± 7.9	11.0 ± 13.6	<0.001
FJS	—	79.1 ± 25.8	80.9 ± 25.1	—	

UKA: unicompartmental knee arthroplasty; KOOS: Knee injury Osteoarthritis Outcome Score; WOMAC: Western Ontario and McMaster Universities Osteoarthritis Score; FJS: Forgotten Joint Score. ^a^Comparison between 5 years and preop.

## Data Availability

Data is available upon request.
